RETRACTED

# Automatic Detection Method of Technical and Tactical Indicators for Table Tennis Based on Trajectory Prediction Using Compensation Fuzzy Neural Network

**DOI:** 10.1155/2021/3155357

**Published:** 2021-08-24

**Authors:** Jin Zhang

**Affiliations:** Department of Public PE Education, Luoyang Normal University, Luoyang, Henan 471934, China

## Abstract

In the system design of table tennis robot, the important influencing factors of automatic detection of technical and tactical indicators for table tennis are table tennis rotation state, trajectory, and rebound force. But the general prediction algorithm cannot process the time series data and give the corresponding rotation state. Therefore, this paper studies the automatic detection method of technical and tactical indicators for table tennis based on the trajectory prediction using the compensation fuzzy neural network. In this paper, the compensation fuzzy neural network algorithm which combines the compensation fuzzy algorithm and recurrent neural network is selected to construct the automatic detection of technical and tactical indicators for table tennis. The experimental results show that the convergence time of the compensation fuzzy neural network is shorter, the training time is shortened, and the prediction accuracy is improved. At the same time, in terms of performance testing, the model can accurately distinguish the influence of table tennis rotation state and rebound on table tennis motion estimation, so as to improve the accuracy of motion trajectory prediction. In addition, the accuracy of trajectory prediction will be improved with the increase of input data. When the number of data reaches 30, the trajectory prediction error is within the actual acceptable error range.

## 1. Introduction

In recent years, with the continuous development and application of big data analysis technology, video technology, and tactics data extraction technology, the pregame auxiliary system has been widely used in the sports industry, which makes the sports industry show significant changes in all aspects [1–4]. The application of these technologies in sports can provide detailed basic data and classified advanced data for athletes and coaches and comprehensively show the advantages and disadvantages of athletes in the competition [5, 6] so that athletes find their own shortcomings and problems and further targeted training. In addition, these data statistics can also predict the results of the competition according to the relevant data of athletes or analyze the changes of competition tactics [7–9]. These detailed data results are generated on the basis of strong computing power, so in the early application of sports data statistics, the data category is less, mainly relying on manual statistics for data processing. However, manual statistics not only requires relevant personnel to have corresponding data analysis ability but also has high error rate and low work efficiency in data processing results [10–12]. With the development of sports industry, the early data analysis can no longer meet the needs of sports development, so the data analysis tool with mature and stable video analysis ability and automatic generation of corresponding technical data has become the key direction of research [13–15]. With the development and maturity of computer vision technology, it has become an important driving force for the scientific and intelligent development of sports industry.

RETRACTED

Table tennis is one of the key sports in China. Due to various reasons, the commercialization level of table tennis is lower than that of basketball and football. Therefore, the application of data statistics with mature technology in table tennis is relatively less [13, 16, 17]. At the same time, in table tennis competition, table tennis has a faster speed and its size is much smaller than basketball and football. Therefore, the data system is difficult to provide accurate information in the speed and rotation direction of table tennis, which improves the difficulty of table tennis positioning and tracking. In addition, in table tennis, table tennis robot research has a very important position, and an excellent table tennis robot can help athletes improve their table tennis technology more efficiently [18, 19]. This requires the table tennis robot to be able to locate the position of the table tennis ball in a short time, predict its trajectory in time, and select the appropriate and reasonable swing mode [20–23]. Therefore, the table tennis robot needs to accurately and automatically monitor the track of table tennis, that is, based on the position information of time series, it can predict the track of table tennis and the landing point on the table and can make the corresponding processing methods in real time [13, 24].

The contributions of this paper are as follows. (1) In view of the above problems, this paper puts forward the research on the automatic detection method of table tennis technical and tactical indexes based on the trajectory prediction algorithm of the compensated fuzzy neural network. (2) Different from the previous table tennis trajectory prediction methods, the compensated fuzzy neural network used in this paper is a hybrid system, which has both the advantages of compensated fuzzy logic and the advantages of the neural network. It has better network fault tolerance and system stability. (3) The method can improve the accuracy of table tennis trajectory prediction and rotation classification. This paper is mainly divided into three parts. The first part introduces the development of automatic detection methods of table tennis technical and tactical indicators and introduces the related concepts. The second part is to construct the automatic detection model of table tennis technical and tactical indexes based on the trajectory prediction algorithm of the compensated fuzzy neural network. The third part analyzes the test data and results of the automatic detection model of table tennis technical and tactical indexes based on the trajectory prediction algorithm of the compensated fuzzy neural network.

RETRACTED

## 2. Related Work

At present, the video data analysis systems in sports and competitions include Hawkeye system applied in tennis competitions and Sport Vu system applied in Western professional basketball competitions. These systems not only collect a large number of relevant data during the competition but also provide reliable visual data analysis and daily training data analysis for athletes and coaches [25]. At the same time, these data analysis systems improve the visibility of live broadcast technology review and greatly improve the audience's viewing experience. Therefore, the automatic detection system of technical and tactical indicators for table tennis has become the research focus of researchers. Many scholars have developed a table tennis robot that can play with people through the combination of a variety of technologies [26]. The relationship between table tennis rotation and table tennis trajectory is also the key research content in the field of table tennis robot control. Some scholars assume that there is a linear relationship between the velocity in two directions parallel to the contact plane and the velocity before and after the collision of the table tennis, obtain the velocity of the table tennis after the collision through the elastic coefficient of restitution, and then predict the trajectory of the table tennis after the collision according to the force situation of the table tennis and the corresponding physical model [27]. In this way, the table tennis trajectory can be predicted in a short time, but the uncertainty of its parameters makes its accuracy low. Some scholars also proposed the influence of Magnus force on the trajectory of table tennis with rotation and, on this basis, constructed a classifier to predict the trajectory based on the BP neural network algorithm. Although in a certain way, the system can distinguish whether the table tennis is in the state of rotation, but it can distinguish the types of rotation is relatively simple, and there is not enough relevant data, and there is a large error. In addition, some scholars have proposed a new way to solve the problem of calculating the rotation of table tennis without special marks. The main idea is to accurately identify the trademark on the table tennis and calculate the rotation direction and the corresponding rotation speed of the table tennis through the movement track of the trademark. In addition, some scholars have designed controllers or control plates for table tennis robots to improve the robot's ability to return the ball. Or, on the basis of empirical data, the algorithm is optimized to obtain the optimal return speed of table tennis robot. Such a table tennis robot has online learning performance, and its return effect will continue to improve with the accumulation of experience data. But its dependence on the accuracy of empirical data is too high, which is easy to cause large errors.

RETRACTED

### 2.1. Construction of Table Tennis Technology and Tactics Index Automatic Detection Model Based on Compensation Fuzzy Neural Network Trajectory Prediction

As shown in Figure 1, it is the framework of this paper. Firstly, the corresponding captured pictures are obtained through the camera module. The detection module is mainly responsible for judging whether the target exists in the picture and outputting the bounding box coordinates. When the detection module does not find the target to be detected, the information is fed back to the camera module and requests to obtain the next frame of picture.

When the detection module detects the corresponding target, the bounding box coordinates are initialized and input into the tracking trajectory prediction algorithm, and then, the algorithm will continuously update and predict the output coordinates. If the tracking trajectory prediction is successful, the corresponding coordinates are output and the motion analysis and visualization module are carried out. Otherwise, the image detection module needs to be adjusted. As shown in Figure 2, the process and optimal results of target detection in the image by the camera and the detection module are shown.

When the table tennis and the racket collide with each other in the movement, in addition to the force produced by the smooth surface contact, there is also the generation of friction, so the resultant force of the table tennis and its center of gravity deviation. The table tennis itself is light in weight and small in volume, and the centrifugal friction generated in the movement will make it rotate faster, resulting in the change of its whole movement trajectory [25]. If we want to predict the impact point and trajectory of table tennis, we need to obtain the relationship between the rotation and trajectory of table tennis by calculation. In order to understand the track and rotation law of table tennis conveniently and intuitively, this paper constructs the world coordinate system and table tennis movement coordinate system, as shown in Figure 3.

RETRACTED

### 2.2. Table Tennis Technology and Tactics Index Automatic Detection Model on Table Tennis Rotation Classification and Influence

The rotation type of table tennis can be analyzed according to its trajectory coordinate system. If table tennis rotates around the *x*-axis in the motion coordinate system, it can be divided into spin ball and counter spin ball according to its rotation direction. If the table tennis revolves around the *y*-axis in the motion coordinate system, it can be divided into downward rotation (clockwise rotation) and upward rotation (counterclockwise rotation) according to its rotation direction. If the table tennis revolves around the *Z*-axis in the motion coordinate system, the rotation direction can be divided into left rotation, that is, clockwise rotation, and right rotation, that is, counterclockwise rotation. But in the actual situation, the rotation of table tennis can make any straight line in the space coordinate system, so when analyzing the rotation of table tennis, we can regard it as the result of the joint action of the three basic coordinate axes of the motion coordinate system and separate it for the corresponding analysis.

If the influence of gravity, air buoyancy, and air resistance on the movement of table tennis is not considered in the process of analyzing the rotation of table tennis, then the pressure balance in all directions around the table tennis is broken and the Magnus force is produced in the process of rotation, and the direction of Magnus force is different with different rotation methods. The results of its influence on table tennis trajectory are also different. Take table tennis left and right rotation as an example to analyze the influence of Magnus force, as shown in Figure 4.

It can be seen from the above figure that when the table tennis is in the left-hand state, the air velocity on the left and right sides is different, and the velocity on the left side is greater than that on the right side. According to Borriel's law, if the air pressure on the left side is less than that on the right side, the Magnus force on the table tennis will be left along the *y*-axis in its motion coordinate system. At this time, the track of *YF* axis is biased to the left and is in the state of positive acceleration, so its speed is constantly improving. Similarly, when the table tennis is in the state of right rotation, the air velocity on the left and right sides is not the same, and the speed on the right side is greater than that on the left side, that is, the air pressure on the right side is smaller; then, the Magnus force on the table tennis is along the *YF* axis to the right, and the track of the *YF* axis is biased to the right and in the state of negative acceleration, so its speed is constantly decreasing. If the table tennis in the state of rotation is analyzed from the change of its velocity and angular velocity, then *ω*=[*ω*_*x*_, *ω*_*y*_, *ω*_*z*_], *v*=[*v*_*x*_, *v*_*y*_, *v*_*z*_] is set, as shown in the following formula:

(1) $$\begin{array}{c} \omega \times v=\left[\omega_{x},\omega_{y},\omega_{z}\right]\times \left[v_{x},v_{y},v_{z}\right]=\left[\omega_{x}v_{z}-v_{y}\omega_{z}\omega_{z}v_{x}-\omega_{x}v_{z}\omega_{x}v_{y}-v_{x}\omega_{y}\right]. \end{array}$$

RETRACTED

### 2.3. Table Tennis Technology and Tactics Index Automatic Detection Model for Table Tennis Trajectory Prediction Algorithm

In the past, when designing the table tennis robot system, the corresponding model was generally built on the basis of CNN (convolution layer neural network) algorithm, but the data processing of the CNN model can only be carried out in the case of single data input [28–31]. In other words, when there is a temporal relationship between the front and back data, the CNN model cannot process the data. The automatic detection system of table tennis technical indicators constructed in this paper needs to solve two problems in table tennis trajectory prediction. On the one hand, the automatic detection system of table tennis technical indicators needs to infer the possible position coordinates of the tracking target at the next moment according to the coordinates of the tracking target at the previous moment. On the other hand, the track prediction of table tennis needs to automatically infer and generate the corresponding coordinate sequence after the known table tennis coordinate sequence data. Therefore, the CNN model cannot solve these two problems, and the recursive compensation fuzzy neural network can meet the needs of these two aspects. The recurrent compensation fuzzy neural network is the combination of the recurrent neural network and compensation fuzzy algorithm. It has both the characteristics of the recurrent neural network and the advantages of the compensation fuzzy algorithm and has good ability to solve the corresponding sequence prediction problems [32–34]. As shown in Figure 5, it is the topology of the recurrent compensation fuzzy neural network.

It can be seen from Figure 3 that most recurrent compensation fuzzy neural networks have multiple input nodes but only one output node, and they have a total of five layers structure, namely, input layer, fuzzification plus recursion layer, fuzzy reasoning layer, rule layer, compensation operation layer, and output layer. If Gaussian function is selected as the membership function of the input variable and output variable, it is shown in following formulas:

(2) $$\begin{array}{c} \mu_{A_{ik}}\left(x\right)=\exp\left[-{\left(\frac{x_{i}-a_{ik}}{c_{ik}}\right)}^{2}\right], \end{array}$$

(3) $$\begin{array}{c} \mu_{B_{k}}\left(y\right)=\exp\left[-{\left(\frac{y-b_{k}}{d_{k}}\right)}^{2}\right]. \end{array}$$

The center of the membership function of the input variable is *a*_*ik*_, and the width is *c*_*ik*_. The center of the membership function of the output variable is expressed as *b*_*k*_, and the width is expressed as *d*_*k*_. If *f*_*i*_^(*q*)^ is used to represent the input of *i* node in *q* layer, *x*_*i*_^(*q*)^ is the output of the node, and *g*_*i*_^(*q*)^ is the excitation function or transfer function of *i* neuron in *q* layer, then the node and input vector are directly connected in the input layer of the first layer, as shown in the following formula:

(4) $$\begin{array}{c} x_{i}^{\left(1\right)}\left(k\right)=g_{i}^{\left(1\right)}=f_{i}^{\left(1\right)}=x_{i}\left(k\right), \end{array}$$

where the number of nodes is *i*=1,2,…, *n* and the corresponding discrete time is *k*; then, *x*_*i*_(*k*) represents the input of *i* node at time *k*.

RETRACTED

In the second layer of fuzzification and recursion, the connection between neurons is not only a forward connection but also a feedback connection, so this layer also has the performance of the memory unit. In the second layer, each node of the neuron has its own input language variable and computes its components. As shown in formulas (5) and (6), the formula is as follows:

(5) $$\begin{array}{c} f_{ij}^{\left(2\right)}\left(k\right)=-{\left(\frac{x_{i}^{\left(1\right)}\left(k\right)+x_{ij}^{\left(2\right)}\left(k-1\right)\circ \theta_{ij}-a_{ij}}{c_{ij}}\right)}^{2}, \end{array}$$

(6) $$\begin{array}{c} x_{ij}^{\left(2\right)}\left(k\right)=g_{ij}^{\left(2\right)}=\mu_{i}^{j}=\exp\left(f_{ij}^{\left(2\right)}\left(k\right)\right). \end{array}$$

Among them, *i*=1,2,…, *n*, *j*=1,2,…, *m*_*i*_, *m*_*i*_ represents the fuzzy partition number of the *i* input, *θ*_*ij*_ represents the weight of feedback connection, *x*_*ij*_^(2)^(*k* − 1) represents the output value of the second layer, and *μ*_*i*_^*j*^ represents the membership between *i* input and *j* language variables.

The nodes in the third fuzzy reasoning layer are mainly used to match the fuzzy rules and calculate the applicability of the rules, as shown in following formulas:

(7) $$\begin{array}{c} f_{j}^{\left(3\right)}=x_{1i_{1}}^{\left(2\right)},x_{2i_{2}}^{\left(2\right)},\ldots ,x_{ni_{n}}^{\left(2\right)}=\mu_{1^{1}}^{i},\mu_{2^{2}}^{i},\ldots ,\mu_{n^{n}}^{i}, \end{array}$$

(8) $$\begin{array}{c} x_{j}^{\left(3\right)}=\alpha_{j}=g_{j}^{\left(3\right)}=f_{j}^{\left(3\right)}, \end{array}$$

in which *i*_1_ ∈ {1,2,…, *m*_1_}, *i*_2_ ∈ {1,2,…, *m*_2_},…, *i*_*n*_ ∈ {1,2,…, *m*_*n*_}, *j*=1,2,…, *m*,  and *m*=∏_*i*=1_^*n*^*m*_*i*_.

RETRACTED

The nodes in the compensation operation layer of the fourth layer are compensation nodes, which mainly carry out the operation of each node's compensation operation, so as to achieve the purpose of dynamically adjusting the fuzzy rules. As shown in formulas (9) and (10), it is the input and output of the fourth layer:

(9) $$\begin{array}{c} f_{j}^{\left(4\right)}={\left[\alpha_{j}\right]}^{1-r_{j}+r_{j}/n}=z_{j}, \end{array}$$

(10) $$\begin{array}{c} x_{j}^{\left(4\right)}=g_{j}^{\left(4\right)}=f_{j}^{\left(4\right)}, \end{array}$$

where *r*_*j*_ is the regulation parameter.

As shown in formulas (11) and (12), it is the formula of the fifth antifuzzifying layer:

(11) $$\begin{array}{c} f^{\left(5\right)}=\frac{\sum_{l=1}^{m}b_{l}d_{l}g_{l}^{\left(4\right)}}{\sum_{l=1}^{m}d_{l}g_{l}^{\left(4\right)}}=\frac{\sum_{l=1}^{m}b_{l}d_{l}z_{l}}{\sum_{l=1}^{m}d_{l}z_{l}}, \end{array}$$

(12) $$\begin{array}{c} y\left(k\right)=x^{\left(5\right)}=g^{\left(5\right)}=f^{\left(5\right)}. \end{array}$$

The center of the membership function to be adjusted is *b*, and its width is *d*; *y*(*k*) is the output value at *k* time.

The training compensation degree is shown in formulas (13)–(15). Let *γ*=(*c*^2^/*c*^2^+*d*^2^),  *γ* ∈ [0,1], and the parameters represented by *c* and *d* can be adjusted:

(13) $$\begin{array}{c} c\left(t+1\right)=c\left(t\right)-\eta \left[\frac{2c\left(t\right)d^{2}\left(t\right)}{{\left[c^{2}\left(t\right)+d^{2}\left(t\right)\right]}^{2}}\right]{\frac{\partial E^{P}}{\partial \gamma }|}_{t}, \end{array}$$

 

(14) $$\begin{array}{c} d\left(t+1\right)=d\left(t\right)+\eta \left[\frac{2c\left(t\right)d^{2}\left(t\right)}{{\left[c^{2}\left(t\right)+d^{2}\left(t\right)\right]}^{2}}\right]{\frac{\partial E^{P}}{\partial \gamma }|}_{t}, \end{array}$$

(15) $$\begin{array}{c} \gamma \left(t+1\right)=\frac{c^{2}\left(t+1\right)}{c^{2}\left(t+1\right)+d^{2}\left(t+1\right)}. \end{array}$$

Among them, *η* stands for learning efficiency.

The cost function of fitting error is shown in following formulas:

(16) $$\begin{array}{c} E=\sum_{P=1}^{P}\sum_{k=1}^{K}E_{k}, \end{array}$$

(17) $$\begin{array}{c} E_{k}=\frac{1}{2}{\left[y_{d}\left(k\right)-y\left(k\right)\right]}^{2}. \end{array}$$

The sample batch is represented as *P*, the final sampling time is represented as *K*, and *y*_*d*_(*k*) represents the actual output at that time, while *y*(*k*) represents the output of the recursive compensation fuzzy model.

RETRACTED

In table tennis trajectory prediction, the *XY* axis of the established coordinate system is suitable for table tennis tables to be parallel to each other and the *Z* axis is perpendicular to the table tennis table. Therefore, the trajectory prediction assumption is only related to the *XY* axis. When the input state is *c*, the probability of the output speed is shown in the following formula:

(18) $$\begin{array}{c} p\left(v|c\right)=\frac{1}{2}\exp\left(-\frac{1}{2}{\left[\begin{array}{c} v_{x}-\mu_{x}\\ v_{y}-\mu_{y}\\ v_{z}-\mu_{z} \end{array}\right]}^{T}{\left[\begin{array}{ccc} \sigma_{x}^{2} & \sigma_{x}\sigma_{y}\rho_{xy} & 0\\ \sigma_{x}\sigma_{y}\rho_{xy} & \sigma_{x}^{2} & 0\\ 0 & 0 & \sigma_{x}^{2} \end{array}\right]}^{-1}\left[\begin{array}{c} v_{x}-\mu_{x}\\ v_{y}-\mu_{y}\\ v_{z}-\mu_{z} \end{array}\right]\right). \end{array}$$

The weight of Gaussian distribution is *k*, and the corresponding probability distribution function is *p*_*k*_. The loss function is shown in the following formula:

(19) $$\begin{array}{c} L\left(v^{*},x\right)=-\log\left(\sum_{k=1}^{K}\theta_{k}\left(c\left(x\right)\right)p_{k}\left(v^{*}|c\left(x\right)\right)\right). \end{array}$$

The output target is represented as *v*^*∗*^, the input of 3D coordinate is represented as *x*, and *c*(*x*) is represented as the intermediate state of the recursive compensation fuzzy model.

## 3. Experimental Results of Table Tennis Technique and Tactics Index Automatic Detection Model Based on Compensation Fuzzy Neural Network Trajectory Prediction Algorithm

### 3.1. Analysis of Training Test Results of Trajectory Prediction Algorithm Based on Compensation Fuzzy Neural Network

This paper is mainly based on the compensation of the fuzzy neural network trajectory prediction algorithm to build table tennis technology and tactics index automatic detection method, and the key problem is the table tennis rotation classification and trajectory prediction. Therefore, the number of fuzzy nodes is 16, the number of fuzzy inference nodes is 54, the number of corresponding compensation nodes is 8, and the accuracy is 0.001. As shown in Figure 6, it is the membership function of the input value without compensation fuzzy neural network training.

The curve shape of the membership function of the compensation fuzzy neural network after training is related to its performance. As shown in Figures 7 and 8, the membership functions of input variables *a* and *b* show the function curves after training. It can be seen from the figure that the center and width of the membership function of the input variable after training have changed.

RETRACTED

Figure 9 shows the training error comparison curve of the compensation fuzzy neural network model and CNN neural network. It can be seen from the figure that the number of iterations required by the compensation fuzzy neural network model to achieve convergence effect and be in a stable state is less than that of CNN neural network model. This shows that the compensation fuzzy neural network has better learning convergence speed, shorter training time, and can judge and predict the rotation state and trajectory of table tennis in a shorter time.

### 3.2. Analysis of Simulation Test Results of Table Tennis Technology and Tactics Index Automatic Detection Model

The automatic detection model of technical and tactical indicators for table tennis firstly selects 330 groups of table tennis related data as the training sample set, as shown in Figure 10, which is the data distribution of various rotation states of table tennis in the training sample.

Figure 11 shows the table tennis technology and tactics index automatic detection model of table tennis rotation state classification results and the actual results of the comparison chart. From the data in the figure, it can be seen that the accuracy of the automatic detection model of technical and tactical indicators for table tennis is high, which basically fits the actual numerical results.

Figure 12 shows the table tennis technology and tactics index automatic detection model of table tennis trajectory prediction test results. From the data and prediction results in the figure, it can be seen that when the number of input coordinates increases, the accuracy of the model is higher. If the input data is in an ideal state, the prediction error of the input data with different lengths will decrease. Especially when the length of input data is 30, the error is less than 40 mm, which is the allowable error range in practical application.

One of the main indexes of table tennis trajectory prediction is the prediction of the next moment position of table tennis. Therefore, this paper carries out the experiment of table tennis technology and tactics index automatic detection model based on the compensation fuzzy neural network trajectory prediction algorithm to predict the next moment position prediction performance, and the results are shown in Figure 13.

When table tennis is in motion, its motion is not just along the parabola trajectory but also needs to consider the situation that the rebound will be produced after the impact between table tennis and the table, and it has an important impact on the prediction of table tennis trajectory. The prediction of the rebound motion of table tennis needs to improve its corresponding weight, and the whole process as long as it changes on the *z*-axis. Because the displacement represented by Gaussian distribution is from the current coordinate position to the next coordinate position of table tennis, that is to say, before the rebound, the velocity on the *z*-axis should be *v* < 0, and after the rebound, it is *v* > 0. It can be seen from Figure 13 that it correctly reflects this situation, that is, before the rebound of table tennis, the mean values of the two Gaussian distributions <0, while after the rebound of table tennis, the mean values of the two Gaussian distributions >0, with smaller sum of standard deviation and higher weight value.

RETRACTED

## 4. Conclusion

With the development and application of science and technology and intelligent technology, it is an important direction of reform and development to improve the data analysis and intelligent level of table tennis. Compared with the traditional manual data analysis, the computer based on big data and video data has better data processing and smaller error algorithm to process the table tennis technical and tactical index data. Therefore, this paper studies the automatic detection method of technical and tactical indicators for table tennis based on the trajectory prediction using the compensation fuzzy neural network. The compensation fuzzy neural network not only has the advantages of the compensation fuzzy algorithm but also has the advantages of the neural network. In other table tennis trajectory prediction algorithms, compensation fuzzy logic is mainly combined with the BP neural network, but the BP neural network will produce large errors in table tennis rotation classification and trajectory prediction due to its own limitations, and it cannot process information with timing. Therefore, this paper selects the combination of the compensation fuzzy algorithm and recurrent neural network to process the time series data, so as to improve the deficiency in time series information processing. The experimental results show that the compensation fuzzy neural network can achieve convergence effect and maintain a stable state in less iterations and has better trajectory prediction effect. In addition, table tennis trajectory prediction has two important factors, one is the rotation state of table tennis, the other is the rebound force of table tennis after hitting the table. Therefore, this paper tests the performance of the table tennis technique and tactics index automatic detection based on the trajectory prediction using the compensation fuzzy neural network. The experimental results show that the automatic detection of technical and tactical indicators for table tennis based on the compensation fuzzy neural network trajectory prediction algorithm can accurately detect and classify the rotation state of table tennis and can detect and correctly reflect the impact of rebound on table tennis trajectory. The final table tennis trajectory prediction test results show that the accuracy of motion trajectory prediction increases with the increase of the number of input data, and when the number of input data reaches 30, the predicted trajectory error is less than 40 mm, which is in line with the error range of practical application. However, the automatic detection method of technical and tactical indicators for table tennis based on the compensation fuzzy neural network trajectory prediction algorithm proposed in this paper still has some shortcomings. There are still large errors in the judgment of the rotation axis of table tennis in the fast rotation, which has an impact on the final table tennis trajectory prediction and will reduce the accuracy of trajectory prediction. With the continuous development and in-depth research of the automatic detection technology of table tennis technical and tactical indicators, table tennis trajectory prediction cannot only improve the viewing of game analysis but also improve the judgment of table tennis robot on table tennis, so as to improve the return quality of table tennis robot and realize the real man-machine game.

RETRACTED

## Figures and Tables

**Figure 1:** The framework of research methods in this paper.

**Figure 2:** The camera and detection module detect the target in the image and the optimal result.

**Figure 3:** World coordinate system and motion coordinate system of table tennis.

**Figure 4:** Air movement when a table tennis ball rotates left-hand.

**Figure 5:** Topology of the recursive compensation fuzzy neural network.

**Figure 6:** Membership function of input values that have not been trained by compensating the fuzzy neural network.

**Figure 7:** The membership function curve of input variable *A* after training.

**Figure 8:** The membership function curve of input variable *B* after training.

**Figure 9:** Contrast curve of training error between the compensating fuzzy neural network model and CNN neural network.

**Figure 10:** The data distribution of various rotation states of table tennis in training samples.

**Figure 11:** Comparison between the classification results of the table tennis rotation state by the automatic detection model of table tennis skills and tactics and the actual results.

RETRACTED

**Figure 12:** Test results of table tennis movement trajectory prediction by the automatic detection model of table tennis technique and tactics index. (a) The predication results when 30 coordinates are entered. (b) The predication results when 5 coordinates are entered.

**Figure 13:** MDN internal state in the rebound process of ping-pong ball. (a) The output of the MDN before rebounding. (b) Output of MDN after rebound.

## Data Availability

The data used to support the findings of this study are available from the corresponding author upon request.
